# Randomized controlled trial testing weight loss and abdominal obesity outcomes of moxibustion

**DOI:** 10.1186/s12938-018-0571-8

**Published:** 2018-11-06

**Authors:** Ching-Hsiu Hsieh, Chi-Chuan Tseng, Ju-Yu Shen, Pei-Ying Chuang

**Affiliations:** 1 Department of Nursing, Chang Gung University of Science and Technology, ChiayiCampus: 2, Chia-pu Rd, West Sec. Pu-tz, 613 Chia-Yi, Taiwan; 2 Department of Traditional Chinese Medicine Chang, Gung Memorial Hospital, Chia-Yi, Taiwan; 3 Department of Early Childhood Educare, Tainan University of Technology, Tainan, Taiwan; 4 School of Nursing, University of Maryland School of Nursing, Baltimore, MD USA

**Keywords:** Moxibustion therapy, Weight reduction, Waist circumference, Waist-to-hip ratio

## Abstract

**Background:**

The purpose of this study was to investigate the efficacy of moxibustion therapy on weight loss, waist circumference and waist-to-hip ratio in young adult females. An experimental design, 51 Asian females were enrolled. Inclusion criteria included females with ages between 21 and 25 years-old and waist circumference ≥ 80 cm, and the exclusion criteria included intolerance to moxibustion therapy and current illness. Two groups were formed, and the subjects in the experimental group received moxibustion sessions lasting 20 min and an educational video program for 30 min; however, participants in the control group received only the educational program every other week for 8 weeks. Dependent variable measurements (e.g., body weight, waist circumference and waist-to-hip ratio) were collected at baseline and follow-up for 8 weeks.

**Results:**

Average body weight of the treatment group decreased significantly from − 1.478 kg (p < 0.0001), while the average body weight in the control group did not decrease significantly − 0.038 kg (p = 0.7197). Also, individuals in the moxibustion experimental group showed significant reductions (p < 0.0001) in both waist circumference and waist-to-hip ratio.

**Conclusion:**

Positive effects on anthropometry can be achieved by moxibustion intervention in conjunction with a weight loss education program. Especially waist circumference and waist-to-hip ratio had more clinically significant and more pronounced for health reasons Future studies can focus on the functional assessment of biomarkers associated with the immune system and relevant mechanisms of action.

## Background

According to the World Health Organization (WHO, 2013), more than 1.4 billion adults were overweight, and over 200 million men and nearly 30 million women were obese in 2008 [1]. Sixty-five percent of the world population lives in countries where excess weight is a larger threat to health than being underweight [2]. Overweight refers to excessive body weight such that the body mass index (BMI; kg/m^2^) is ≥ 25, while obesity refers to a BMI ≥ 30 [3]. These standards for excess weight are commonly used in the US, Europe and Australia. The Centers for Disease Control and Prevention (CDC), the National Health and Nutrition Examination Survey (NHANES) and the National Health Interview Survey (NHIS) report that 6.3% of males and 8% of females 20 years of age and older have BMI values of 40 or higher and classify as extremely obese [4–6]. These critical global health issues have raised the attention of healthcare providers and are also recognized to be potentially harmful to younger generations.

Excess weight can be assessed through measures other than BMI. For example, abdominal obesity, which is more common among men (who tend to have an android body fat distribution) than women (who tend to accumulate fat around the hips and thighs in a gynoid distribution), is another parameter that can be examined to study weight. The two most common ways to measure abdominal obesity are through waist circumference (WC) and by comparing waist size to hip size (waist-to-hip ratio, WHR). WC is an anthropometric index commonly used as a proxy for abdominal fat mass [7, 8], which is calculated by placing a measuring tape around the abdomen at a horizontal level just above the hip bone. According to the classifications adopted by the American Heart Association and the National Heart, Lung, and Blood Institute of the US National Institutes of Health, elevated WC is defined as ≥ 102 cm in males and as ≥ 88 cm in females [9, 10]. Multiple prospective cohort research studies have shown that a relationship exists between abdominal obesity (assessed both by WC and WHR) and subclinical atherosclerotic vascular disease regardless of race, sex or age group [11]. In particular, Lee and colleagues showed that WC and WHR predict coronary artery calcification (CAC) [12–14]. High WC values are also associated with other complications such as metabolic syndrome [11], which is a constellation of metabolic risk factors that negatively affect human health. The most common health consequences associated with excess weight include cardiovascular disease, diabetes, musculoskeletal disorders and several cancer [1].

The total annual cost related to the current prevalence of adolescent excess weight is estimated to be $254 billion in the US and €59 billion in the EU member states. Certainly, the ramifications of this global epidemic include limitations to the daily physical activities of individuals with excess weight and also an increased economic burden [9, 15] Childhood rates of excess weight continue to increase; therefore, effective interventions that can be employed as early as infancy to reverse the anticipated trends and the identification of efficacious methods to treat excess weight in younger individuals are necessary to combat this global health problem [7].

Two popular alternative medicine treatments, acupuncture and moxibustion, arose from traditional Chinese medicine and share the following three similar principles: (1) modification of central nervous system neurotransmitter levels through repeated acupoint stimulation; (2) enhancement of the immune system; and (3) channel point stimulation [16–20]. However, moxibustion uses moxa to warm body regions and acupoints by stimulating circulation and by inducing a smoother flow of blood and qi [4, 17–21]. Moxibustion can be applied to patients directly (burn cones up to 1 cm in size are placed directly onto the skin) or indirectly (a medium is placed in between the burning moxa and the skin). Moxibustion may be a good alternative for patients who want to avoid skin penetration during acupuncture. As detailed in Chinese medical books, 361 channel points can be used to assess pathological changes to help diagnose disease [22–24].

Moxibustion interventions have been studied in both animal and human models. Several studies in animal models have demonstrated the positive effects of moxibustion in females with excess body weight and endocrine issues. For example, Zhu and colleagues found that preventive moxibustion had beneficial effects on fat accumulation, blood lipids, and estradiol (E2) levels in menopausal rats [24]. Specifically, Zhu and colleagues found that total plasma cholesterol decreased and the rate of body weight gain was slowed in the moxibustion treatment group compared with the control group in 14-month-old rats. These findings suggest that moxibustion has beneficial effects on both blood lipids and body weight management. Spleen and thoracic gland function indices have also been measured as well as synoviocytes collected from knee joints. Overall, these results have shown that moxibustion has a positive impact on the pathological pathways of the immune system [25, 26].

Other studies have shown that moxibustion has positive effects on human health. For example, a Chinese research study showed that polycystic ovary syndrome is strongly correlated with obesity and insulin resistance in women. Women with these symptoms who were treated with moxibustion displayed increased adiponectin expression, a protein associated with improved insulin sensitivity [26]. Another relevant study examined the effects of moxibustion treatment over 3 months in 150 Chinese women with climacteric syndrome. The points chosen for treatment were Quchi (LI 11), Zhongwan (CV 12), Tianshu (ST 25), Daheng (SP 15), Zusanli (ST 36), Shangjuxu (ST 37), Sanyinjiao (SP 6) and Neiting (ST 44), and an intense moxibustion intervention was employed (i.e., the subjects were treated every other day for 3 months). The outcome variables [e.g., symptoms, physical signs, obesity index, Kupperman index, the vegetative equilibrium index (value Y), estradiol (E2) and follicle stimulating hormone (FSH)] were assessed before and after treatment. Significant reductions in the obesity index, Kupperman index, and FSH levels were observed after moxibustion treatment. The authors concluded that deficiencies in liver, spleen and kidney function may be associated with climacteric syndrome and should be closely monitored in obese individuals who are at risk for this syndrome [27]. To date, researchers have reported that moxibustion has worked on several populations such as obese females with climacteric syndrome and polycystic ovary syndrome, gastric mucosal injury, weight gain/loss, short stature, kidney deficiency in children, and partial androgen deficiency in males [25–32].

A variety of treatments for excess weight exist, including changing lifestyle habits such as dietary and physical activity patterns and other behavioral changes as well as weight-loss medicines and surgeries. Furthermore, alternative medicine treatments for excess weight are becoming increasingly popular. For example, in the US, moxibustion/acupuncture, massage therapy, meditation, movement relaxation techniques, spinal manipulation, and Tai Chi were among the top ten most commonly used alternative medicine treatments in 2007 [16, 33–35].

This study was to investigate the efficacy of moxibustion therapy on weight loss, waist circumference and waist-to-hip ratio in young adult females.

## Methods

### Demographics and study design

An experimental design was used to test the effects of indirect moxibustion on weight loss and abdominal obesity. Sixty participants were recruited from a private university in Taiwan and were assigned randomly by a computer-generated list to one of two groups (control or experimental). The randomization was confidential, and no one except the principal investigator knew the treatment allocation of the patients. The inclusion criteria included the following: (1) age 21–25 years-old; (2) Asian female; and (3) WC ≥ 80 cm, which is deemed excessive for Asian females by the Bureau of Health Promotion, Department of Health, R.O.C. (Taiwan) [36]. The exclusion criteria included the following: (1) medication allergies; (2) present illness (e.g., cold or flu); and (3) moxibustion intolerance.

Demographic data were collected at the first visit. The ethics committee approval was obtained from Chang Gung Medical Foundation Institutional Review Board (100-2867A3), and informed consent was obtained from each participant and informed consent was obtained from each participant. All participants had the right to withdraw from the study at any time. No potential harm or risk from participating in the study was expected or reported. The potential benefits of participation in the study were weight loss, improved health and increased overall wellbeing.

A diet and daily activity education program was designed for each participant. Group A (the control group) received the educational program, and group B (the experimental group) received both the educational program and moxibustion treatment. Framework of the study (Fig. 1). The educational program involved a 30-min video detailing healthy habits focused on reduced-calorie diets and lifestyle modification techniques. The programs were given at separate times to reduce bias. After watching the educational video, all participants were allowed to ask questions regarding the video program, which were answered by a senior nurse who was familiar with the video. Body weight (BW), WC, and WHR were recorded for all participants every 2 weeks (four total times) throughout the study.

**Fig. 1:** A flow chart of the study design

In the experimental group, each participant received 20 min of indirect moxibuston twice a week for a total of 8 weeks. The acupoints targeting weight loss were the Guanyuan (RN4), Qihai (RN6), Shuifen (RN9), Xiawan (RN10) and Tianshu (ST25) points. A senior Chinese medical practitioner lit one end of a moxa stick (approximately 20 cm in length, roughly the shape and size of a cigar) and held the stick close to the area being treated for 20 min until the skin turned light pink and warm. After this desired effect was achieved, the moxa was extinguished, and the practitioner briefly checked the pulse of the participant.

## Results

During the 8 weeks of the study, 9 participants withdrew for a variety of reasons such as generally feeling uncomfortable with traditional Chinese medicine and disliking the sensation of the burning moxibustion (experimental group, n = 3) and the inability to follow the treatment schedule (control group, n = 4; experimental group, n = 2), and these 9 subjects are not included in the final analysis.

The data were analyzed using SPSS software (SPSS 19.0. for Windows).Mean and standard deviations of BW, WC and WHR score were compared among subjects who were treated with moxibustion plus education or education only. In the primary study outcome measures of differences between both groups were analyzed using linear mixed model analysis of variance with group and meeting time as fixed effects for continuous outcomes. Normally distributed variables and generalized estimating equations for categorical variables.

Twenty-five (49%) subjects were included in the moxibustion treatment group (B), and twenty-six (51%) subjects were in the control group (A). Those anthropometrics are different between two groups. The differences are significant in body weight (BW) (p = 0.002) and waist circumference (WC) (p = 0.003). The anthropometric characteristics of the participants at baseline are reported in Table 1.

**Table 1:** Baseline anthropometrics of the two groups (n = 51) expressed as the mean ± standard deviations (SD)

	Mean ± SD		p-value^a^
	Control (n = 26; 51%)	Experimental (n = 25; 49%)	
BW (kg)	67.66 ± 14.45	54.10 ± 8.34	0.0002
WC (cm)	85.71 ± 10.83	74.83 ± 8.90	0.0003
WHR	0.8452 ± 0.056	0.8150 ± 0.055	0.0575

^a^From comparison between control and experiment groups using group-t-test

During the 8 weeks of treatment, three major outcome variables (BW, WC, and WHR) were monitored in both groups. Tables 2, 3 and 4 present the change. So the difference between follow-up and baseline were calculated at teach week (follow-up–baseline). Then mean and SD of those differences to show anthropometrics changed with the intervention time. The test between each follow-up week and baseline was performed. Also the mean changed at each week was compared between two groups. The trend of change with time (slope) was also looked at by fitting a linear model with a mixed model for each group, and compared between groups. In the control group, the females did not show a significant overall change in BW (− 0.038 ± 0.540 kg; *p *= 0.7197 at week 8); however, WC (0.673 ± 1.655 cm; *p *= 0.0485 at week 8) and WHR (0.003 ± 0.014; *p *= 0.1163 at week 8) were elevated, indicating a trend of increasing size in these individuals. In contrast, the participants who received moxibustion therapy were noted to have continual losses in BW (− 1.478 ± 1.075 kg at week 8; *p* < 0.0001) (Table 2). For the control group, the changes in BW (mean ± SD) during intervention were not significant (p > 0.05), and the slope with time was not significant (p = 0.0961), however, BW is decreased during follow-up slightly. In the experiment group, BW (mean) decreased with time, and the change is − 0.212 at week 2, − 0.728 at week 4, − 1.039 are week 6 and − 1.478 at week 8. The slope with time is very significant (p < 0.0001). The comparisons between groups in mean at different week are not significant until week 6 and overall slope is very significant between two groups.

**Table 2:** Changes in BW over the 8-week intervention program

Week	Control group (kg), mean ± SD	p-value^a^	Experimental group (kg), mean ± SD	p-value^a^	p-value^b^
	(n = 26)		(n = 25)		
1st week	0		0		
2nd week	0.142 ± 0.489	0.1505	− 0.212 ± 0.357	0.0067	0.0050
4th week	0.077 ± 0.418	0.3580	− 0.728 ± 0.587	< 0.0001	< 0.0001
6th week	0.069 ± 0.562	0.5356	− 1.039 ± 0.712	< 0.0001	< 0.0001
8th week	− 0.038 ± 0.540	0.7197	− 1.478 ± 1.075	< 0.0001	< 0.0001
Slope of time (SE)	− 0.0134 (0.008)	0.0961	− 0.1939	< 0.0001	< 0.0001

^a^p-value: from comparison between each week during the follow-up and the baseline measure (week 1)

^b^p-value: from comparison between control and experiment groups

**Table 3:** Changes in waist circumference (WC) over the 8-week intervention program

Week	Control group (kg), mean ± SD	p-value^a^	Experimental group (kg), mean ± SD	p-value^a^	p-value^b^
	(n = 26)		(n = 25)		
1st week	0		0		
2nd week	0.365 ± 1.054	0.0894	− 0.471 ± 1.165	0.0544	0.0097
4th week	0.577 ± 1.181	0.0197	− 1.710 ± 2.013	0.0003	< 0.0001
6th week	0.712 ± 1.733	0.0466	− 2.499 ± 2.542	0.0001	< 0.0001
8th week	0.673 ± 1.655	0.0485	− 3.157 ± 3.289	0.0001	< 0.0001
Slope of time	0.0798	0.0003	− 0.4240	< 0.0001	< 0.0001

^a^p-value: from comparison between each week during the follow-up and the baseline measure (week 1)

^b^p-value: from comparison between control and experiment groups

**Table 4:** Changes in waist size to hip size (waist-to-hip ratio, WHR) over the 8-week intervention program

Week	Control group (kg), mean ± SD	p-value^a^	Experimental group (kg), mean ± SD	p-value^a^	p-value^b^
	(n = 26)		(n = 25)		
1st week	0		0		
2nd week	0.001 ± 0.011	0.7269	− 0.001 ± 0.018	0.8044	0.6942
4th week	0.004 ± 0.012	0.1092	− 0.007 ± 0.025	0.1813	0.0596
6th week	0.006 ± 0.016	0.0717	− 0.014 ± 0.027	0.0212	0.0040
8th week	0.003 ± 0.014	0.1163	− 0.019 ± 0.028	0.0045	0.0019
Slope of time (SE)	0.0007	0.0046	− 0.0023	< 0.0001	< 0.0001

Change was calculated as follow-up measurement minus baseline measurement (week 1)

^a^p-value: from comparison between each week during the follow-up and the baseline measure (week 1)

^b^p-value: from comparison between control and experiment groups

WC (− 3.157 ± 3.289 cm at week 8; p < 0.0001) (Table 3). For the control group, the changes in WC during intervention are significant (p < 0.05) except at week 1 and the slope with time is also significant (p = 0.0003), suggesting WC is increased with time. In the experiment group, WC decreased with time, and the change is − 0.471 at week 2, − 1.710 at week 4, − 2.499 are week 6 and − 3.157 at week 8. The slope with time is very significant (p < 0.0001). The comparisons between groups in mean at different week or slopes are all very significant. WHR (− 0.019 ± 0.028 at week 8; p < 0.0001). For the control group, the changes in WHR during intervention are not significant (p > 0.05), but the slope with time is significant (p = 0.0046), suggesting WHR is increased during follow-up slightly. In the experiment group, WHR decreased with time, and the change is − 0.001 at week 2, − 0.007 at week 4, − 0.014 are week 6 and − 0.019 at week 8. The slope with time is very significant (p < 0.0001). The comparisons between groups in mean at different week are not significant until week 6 and overall slope is very significant between two groups (Table 4). Thus, the moxibustion therapy in conjunction with the weight loss education program led to decreased body weight in this study.

Furthermore, we also administered a short questionnaire on the educational program and moxibustion therapy to all participants. This questionnaire identified several potential intervention areas that can be applied to future research strategies. For example, 13 responders recommended that healthy, low-calorie recipes be provided to facilitate the adoption of the lifestyle changes suggested in the program. Five responders suggested extending the follow-up moxibustion therapy to 6 months. Their feedback and comments were based on their positive experiences with the moxibustion therapy administered over the study period of 2 months. Four participants shared their experience that a meet-up support group may be an effective method to continually motivate people to prioritize their health and body image.

## Discussion

In the current study, 8 weeks of moxibustion therapy with a weight loss education program significantly decreased participant BW, WC and WHR. The weight loss finding is supported by another study that assessed the efficacy of acupuncture treatment on weight over 3 months and showed significant weight loss (*p *< 0.05) in the treatment group [37]. An additional study that treated 100 obese patients with acupuncture for 30 days also reported significant mean weight loss (*p *< 0.05) [35]. Beyond weight loss effects, acupuncture point stimulation has been shown to have additional benefits to anthropometry. A different study by our group found that ear acupressure administered for 8 weeks decreased BW, WC and WHR [38]. Similarly, Lien and colleagues showed that auricular stimulation over 4 weeks decreased BW, WC and WHR [21].

This study has several limitations. The sample size was small and only included females. Additionally, we did not collect detailed demographic characteristics or perform clinical laboratory tests. In future studies, we will seek to increase the sample size, include males, and investigate personal and family health histories (e.g., cardiovascular disease, kidney disease, diabetes, and several cancers associated with excess weight). We will also perform laboratory tests (e.g., cholesterol and low and high density lipoproteins) to better understand the physiological effects of moxibustion. Studies involving long-term treatment as well as follow-up after treatment will also be important considerations for future studies. Furthermore, comparisons between moxibustion and acupuncture should be performed to assess their efficacy in treating body fat in specific regions such as the upper arms, abdomen, thighs and lower legs. Lastly, future studies should focus on elucidating the mechanisms by which moxibustion treatment affects body composition. However, Study design had major weaknesses: (a) There was no sham treatment, which made it might impossible to interpret the result—the small effects might have been simple placebo. The controls received one training session at the beginning and no other intervention apart from bi-weekly weighing, while the moxibustion group received twice weekly moxibustion treatments. (b) An average person’s weight fluctuates more than that over the course of a day, and considerably larger variations might normal over the course of the menstrual cycle in women. Those are also be important considerations for future studies.

## Conclusion

This study showed that moxibustion therapy in parallel with a weight loss education program decreases BW, WC and WHR in Asian females after 8 weeks of treatment. These results suggest that moxibustion may offer an effective and economical treatment for excess weight that can be used in addition to more conventional treatments such as exercise, diet control, medicine and surgery. After calculating the statistics, (treatment group lost a mean of − 1.478 kg over 8 weeks), although the weight numbers are still tiny but statistically significant. Also, the numbers throughout the study showed that changes in waist circumference: − 3.157 cm is more clinically significant and more pronounced in waist-to-hip changes for health reasons. There is no single cause for excess weight; therefore, there is no single approach that prevents or treats excess weight. Diet, exercise, and lifestyle choices are the cornerstone of weight management; moxibustion may be an effective supplemental treatment.
